The article "Immunoglobulin G Expression in Lung Cancer and Its Effects on Metastasis" was retracted in 2020. Reasons: duplicated images; concerns about the results or conclusions.

# Immunoglobulin G Expression in Lung Cancer and Its Effects on Metastasis

**DOI:** 10.1371/journal.pone.0097359

**Published:** 2014-05-22

**Authors:** Chunfan Jiang, Tao Huang, Yun Wang, Guowei Huang, Xia Wan, Jiang Gu

**Affiliations:** 1 Guangdong Provincial Key Laboratory of Infectious Diseases and Molecular Immunopathology, Department of Pathology, Shantou University Medical College, Shantou, Guangdong, China; 2 Department of pathology, Xiangyang Central Hospital, Affiliated Hospital of Hubei University of Arts and Science, Xiangyang, Hubei, China; 3 Translational Medicine Center, Second Affiliated Hospital, Shantou University Medical College, Shantou, China; Kliniken der Stadt Köln gGmbH, Germany

## Abstract

Lung cancer is one of the leading malignancies worldwide, but the regulatory mechanism of its growth and metastasis is still poorly understood. We investigated the possible expression of immunoglobulin G (IgG) genes in squamous cell carcinomas and adenocarcinomas of the lung and related cancer cell lines. Abundant mRNA of IgG and essential enzymes for IgG synthesis, recombination activation genes 1, 2 (RAG1, 2) and activation-induced cytidine deaminase (AID) were detected in the cancer cells but not in adjacent normal lung tissue or normal lung epithelial cell line. The extents of IgG expression in 86 lung cancers were found to associate with clinical stage, pathological grade and lymph node metastasis. We found that knockdown of IgG with siRNA resulted in decreases of cellular proliferation, migration and attachment for cultured lung cancer cells. Metastasis-associated gene 1 (MTA1) appeared to be co-expressed with IgG in lung cancer cells. Statistical analysis showed that the rate of IgG expression was significantly correlated to that of MTA1 and to lymph node metastases. Inhibition of MTA1 gene expression with siRNA also led to decreases of cellular migration and attachment for cultured lung cancer cells. These evidences suggested that inhibition of cancer migration and attachment induced by IgG down-regulation might be achieved through MTA1 regulatory pathway. Our findings suggest that lung cancer-produced IgG is likely to play an important role in cancer growth and metastasis with significant clinical implications.

## Introduction

Lung cancer is one of the leading malignant tumors worldwide with a very high mortality [1], [2]. Metastasis is the main cause of death and up to date there is no effective treatment to metastatic lung cancer. Lung cancer can be divided into non-small cell lung cancer (NSCLC) and small cell lung cancer (SCLC) based on their pathological features and clinical behavior [3]. NSCLC accounts for 84% of lung cancers, of which the majority are squamous cell carcinoma (LSCC) and adenocarcinoma (LAC) [4]. LSCC and LAC were chosen as the objects of this study.

The article "Immunoglobulin G Expression in Lung Cancer and Its Effects on Metastasis" was retracted in 2020. Reasons: duplicated images; concerns about the results or conclusions.

Recently, cumulative evidences have shown that human tumor cells including cancers of breast, lung, prostate, colon, esophagus, thyroid and placental trophablast as well as sarcomas can synthesize immunoglobulin G (IgG) [5]–[19]. The essential enzymes including recombination activation genes 1, 2 (RAG1, 2) and activation-induced cytidine deaminase (AID) for synthesizing IgG in B lymphocytes and plasma cells were also found in cancer cells [20]–[22]. CA215, an immunoglobulin superfamily protein initially isolated from ovarian cancer was thought to be the IgG of cancerous origin [23]–[25]. Blockade of cancerous IgG with antisense RNA or IgG antibody suppressed cancer cell growth and increased apoptosis [5], [26]–[28]. By detecting IgG expression in 142 esophagus cancers and 80 soft tissue tumors, and comparative analysis of IgG expression with pathological parameters, cancerous IgG was found to correlate with tumor grade and proliferative markers such as PCNA and ki-67 in cancers of the breast, esophagus and soft tissues [8], [11], [29]. These results suggest that cancerous IgG might play a role in regulating cancer growth. However, the effect of IgG in lung cancer and the possible mechanism governing its actions have not been investigated.

Metastasis is a complex process involving various proteins that act on detaching cancer cells from primary sites, infiltrating into vessels and lymphatics, anchoring to endothelia, intruding into surrounding matrix, extravasating, inducing angiogenesis, avoiding anti-tumor immunity, and growing at metastatic sites. Metastasis-associated gene 1 (MTA1) is an integral part of the nucleosome remodeling and deacetylating (NuRD) complex of histone [30], [31]. MTA1 regulates the transcription of metastasis related genes by modifying the target chromatin acetylation status as well as cofactor accessibility to the target DNA. High MTA1 expression has been found to be closely related to invasion and lymphatic metastasis in various carcinomas [32]–[34].

In this study, we examined the distribution pattern of IgG, and the relationship between its expression and pathological parameters in 86 LSCC and LAC. We further investigated the possible effects of cancer-produced IgG on cellular attachment and migration by using the technique of siRNA interference in an attachment assay, a transwell assay, and a wound healing assay with two lung cancer cell lines as well as a normal lung epithelial cell line. We also studied the relationship between IgG gene expression and a number of metastatic related genes. We found that cancerous IgG may play a key role in lung cancer metastasis through regulating the metastatic gene MTA1.

The article "Immunoglobulin G Expression in Lung Cancer and Its Effects on Metastasis" was retracted in 2020. Reasons: duplicated images; concerns about the results or conclusions.

## Materials and Methods

### Ethics statement

This study was carried out in accordance with the Helsinki Declaration and approved by the Ethical Committee of Shantou University Medical College. Written informed consent was obtained from patients or their families for using the specimens for research.

### Cell lines

Human lung squamous cell carcinoma cell line SK-MES-1, lung adenocarcinoma cell line A549, normal lung epithelial cell line Beas2B, and Burkitt's lymphoma cell line Raji were purchased from ATCC (Manassas, VA, US) and cultured in DMEM with 10% FBS. All the cell lines were cultured in humidified atmosphere with 5% CO_2_ at 37°C.

### Tissue samples

Eighty-six formalin fixation paraffin embedded lung cancer specimens including adjacent normal lung tissue were retrieved from Department of Pathology, Shantou University Medical College affiliated Tumor Hospital and Department of Pathology, Xiangyang Central Hospital, Hubei province from 2006 to 2011 with complete clinical information of ages, sex, histological type, pathological grade, clinical stage and lymph node metastasis. Two practicing pathologists re-examined the hematoxylin and eosin (H&E) slides to verify the diagnosis independently. For immunohistochemistry (IHC) and in situ hybridization (ISH), specimens were cut into 3 µm thick serial sections. Four fresh surgical specimens (two LSCCs and two LACs with adjacent normal tissue) were obtained from Department of Cardiothoracic Surgery, Shantou University Medical College affiliated Tumor Hospital and preserved at −80°C before extracting RNA from cells isolated with laser guided microdissection (LMD).

### Immunohistochemistry

IHC was performed as described previously [35]. Briefly, 3.5 µm sections were deparaffinized in xylene, hydrated in decreasing concentrations of ethanol and then rinsed in running tap water. The slides were incubated with primary antibodies at 4°C overnight. Subsequently, the slides were incubated with a secondary antibody (PV9000; Zymed Laboratory, South San Francisco) and visualized with 3-amino-9-ethyl-carbazole (AEC; Golden Bridge International). The primary antibodies were listed in Table S1. Autopsied healthy tonsil tissues were used as positive controls for Igγ, Igκ and Igλ immunostainings. PBS instead of primary antibodies was used as a negative control. To assure the specificity of immunostaining, an antibody pre-absorption test was performed in which the primary antibody against Igγ was pre-incubated with pure human IgG at the molar ratio of 1∶1, 1∶5 and 1∶10. The mixed solution was incubated at 4°C overnight and then used in place of the primary antibody.

The article "Immunoglobulin G Expression in Lung Cancer and Its Effects on Metastasis" was retracted in 2020. Reasons: duplicated images; concerns about the results or conclusions.

### Igγ and MTA1 expression scoring

Scoring of the Igγ immunostaining was performed as previously described with minor modification [8]. The percentage and intensity of positive cells were acquired by counting tumor cells from 10 randomly selected visual fields under 400×magnification. Scoring of 0–3 for the percentage of positive cells was: 0 = <5%; 1 = 5–25%; 2 = 25–50%; and 3 = >50%. The intensity of IHC staining was scored: 0, 1, 2, 3, representing absence of signal, weak signal (light red), moderate signal (red) and strong signal (dark red), respectively. The final result for each case was determined by adding the two scores together and the overall results were assigned negative (−) when the sum was 0 or 1, weakly positive (+) when the sum was 2 or 3, moderately positive (++) when the sum was 4 or 5, and strongly positive (+++) when the sum was 6. To study the relation between Igγ and MTA1, the samples of lung cancer were divided into 2 groups according to the scores of Igγ immunostaining. Cases with scores of 0–3 were regarded as “weak expression” and 4–6 as “strong expression”.

Scoring of the MTA1 immunostaining was calculated by using a labeling index (LI) as follows: LI  = 100×(p/t)% (“p” is the number of MTA1-positive cancer cells and “t” is the number of total cancer cells). Approximately 3000 cells under ×400 magnification were counted (10 randomly selected fields on each slide).

### In situ hybridization

The probes were designed to detect human immunoglobulin G1 heavy chain constant region (IGHG1). PCR primers for IGHG1 were as follows: sense, 5′-ACGGCGTGGAGGTGCATAATG-3′; antisense, 5′-CGGGAGGCGTGGTCTTGTAGTT-3′. The method to synthesize the specific probes have been reported previously [6]. In short, a ruptured spleen caused by trauma was used to separate lymphocytes. The PCR product was subcloned into pGEM-T vector (Tiangen Biotech, Beijing, China). Subsequently, the endonuclease *Nco*I or *Sal*I was used to linearize the new plasmid, and T7 or Sp6 RNA polymerase was used to generate the antisense or sense probe with the new plasmid as a template.

ISH was performed as previously described [8]. In short, deparaffinized, rehydrated tissue slides were treated with 0.1 M Hcl for 10 min, heated to 100°C in citrate buffer (0.01 M, pH 6.0) for 15 min, fixed in 4% paraformaldehyde for 10 min and then dehydrated by 90% ethanol. Until dry completely, slides were incubated with 20 µl hybridization mix containing 18 µl diluent and 2 µl sense or antisense probe at 50°C for 18∼20 h. After washing with 5×SSC, 2×SSC plus 50% formamide and 2×SSC twice for 15 min at 37°C, slides were blocked with horse serum at room temperature for 1 h, and incubated with anti-digoxigemin-Ap Fab fragments(1∶500, Roche Diagnostics, Rotkreuz, Switzerland) at room temperature for 1 h. Slides were colored by using NBT-BCIP (Promega, Madison, USA). For cultured cells growing on slides, all the procedures were similar to tissue slides except deparaffin, rehydration and heating retrieval. Additional slides were incubated with the sense probes as negative controls.

The article "Immunoglobulin G Expression in Lung Cancer and Its Effects on Metastasis" was retracted in 2020. Reasons: duplicated images; concerns about the results or conclusions.

### Immunofluorescence

A549, SK-MES-1 and Beas2B were allowed to grow on slides. Immunofluorescence was performed according to a protocol as described previously [11]. The primary antibodies used in this assay are described in Table S1. After washing in PBS, slides were incubated with FITC-conjugated goat anti-rabbit/goat anti-mouse IgG (Zhongshan Golden Bridge, Beijing, China) at room temperature for 30 min. DAPI was utilized to counterstain nuclei. The slides were examined and photographed with a fluorescence microscope (Zeiss AxioImager Z1, Zeiss GmbH, Göttingen, Germany).

### Laser guided microdissection, RNA extraction and reverse transcription

Fresh frozen tissue samples were sectioned at 10 µm, mounted on a polyethylene naphthalate (PEN)-membrane slide (Leica Microsystems, Wetzlar, Germany) and then immediately fixed in 75% ethanol for 1 min. Target cells in sections were microdissected and collected to the cap of an Eppendorf tube with laser power using the Leica Microdissection Systems 6000 (Leica Microsystems, Wetzlar, Germany). Total RNA was extracted from isolated cells with a RNeasy Micro Kit (Qiagen, Hilden, Germany). Target cDNAs were synthesized with a superscript III first-strand synthesis kit (Invitrogen, Carlsbad, CA) according to the manufacturer's instructions.

TRIZOL (Invitrogen), chloroform, isopropanol and ethanol were utilized to extract RNA from tissue samples according to a protocol provided by Invitrogen. RNase Free DNase (invitrogen) was utilized to remove possible genomic DNA contamination. Target cDNAs were generated with first strand cDNA systhesis kit (Toyobo scientific, Shanghai, China) according to the manufacturer's instructions.

### Polymerase chain reaction (PCR)

As described previously, IGHG1, RAG1, RAG2, and AID were amplified with nested PCR [8]. The primers (Sangon Biotech, Shanghai, China) used in this assay are listed in Table S2. The PCR products were examined with 2% agarose gel electrophoresis. Water instead of cDNA was used as the PCR templates as negative controls for those genes whose primers span two exons. For RAG1, RAG2 and Igκ, whose primers located in one exon, RNA treated with DNase was used as a negative control. Raji cell line was employed as a positive control. Housekeeping gene GAPDH was used to normalize the relative expression levels.

The article "Immunoglobulin G Expression in Lung Cancer and Its Effects on Metastasis" was retracted in 2020. Reasons: duplicated images; concerns about the results or conclusions.

### DNA sequencing

PCR prodocts for Vγ, Vκ and Vλ were extracted with Agarose Gel DNA Extraction Kit (TaKaRa Biotech, Dalian, China) and then cloned in to a pGEM-T vector (Tiangen Biotech, Beijing, China). After transfected into Competent *E. coli* TOP10, new clones were formed that were amplified with bacteria breeding. Subsequently, new clones were purified with the Universal DNA Purification Kit (Tiangen Biotech) and examined with 2% agarose gel electrophoresis. The new clones were used in DNA sequencing, which was performed by BGI-Shenzhen, China. The sequences of the new clones were compared to known sequences in the GenBank website (http://www.ncbi.nlm.nih.gov/BLAST).

### Real-Time PCR and Quantitative Analysis

Using an ABI PRISM 7500 instrument, real-time PCR was performed with SYBR Premix Ex Taq II (TaKaRa Bio, Inc., Dalian, China) according to manufacturer's instructions. To detect downstream genes possibly regulated by IgG, common metastatic genes MTA1, CD44, E-cadherin, MMP9, MMP2 and Intergrin β1 were examined following siRNA interference (see “RNA interference”). The primers used for real-time PCR are listed in Table S3. Amplification of β-actin was used for normalization. The relative expressions of each gene in the tested cell types were determined with the method of 2^−ΔΔCt^ [36].

### Western blot

Western blot was performed as previously described [11]. Protein aliquots 150 µg was run on 10% sodium dodecyl sulfate-polyacrylamide gel electrophoresis (SDS-PAGE). The whole molecular IgG was on non-reducing gels and other proteins were on reducing gels. The primary antibodies used in this assay are described in Table S1. To detect the downstream genes possibly regulated by IgG, common metastatic genes MTA1, CD44, E-cadherin, MMP9, MMP2 and Intergrin β1 were examined following siRNA interference of IgG genes. Pure human IgG was used as a positive control and housekeeping gene β-actin was used to normalize the relative expression levels.

### RNA interference

The cultured A549, SK-MES-1 and Beas2B cells were divided into three groups (siRNA-IGHG1 or siRNA-MTA1, siRNA-scrambled and the untreated). Scrambled siRNAs were used as a negative control. All the siRNAs were purchased from Shanghai GenePharma Inc. The IGHG1 siRNA sequences were sense: 5′- CCAAGGACACCCUCAUGAUTT-3′ and antisense: 5′-AUCAUGAGGGUGUCCUUGGTT-3′; MTA1 siRNA sequences were sense 5′-GCUGAGAGCAAGUUAAAGCTT-3′ and antisense 5′-GCUUUAACUUGCUCUCAGCTT-3′; scrambled siRNA sequences were sense: 5′-UUCUCCGAACGUGUCACGUTT-3′ and antisense: 5′-ACGUGACACGUUCGGAGAATT-3′. For the siRNA transfection, X-tremeGENE reagent (Roche Diagnostics) was used. The ratio of transfection reagent to siRNA was 10 µl: 2 µg per 3×10^5^ cells. The transfection procedure was carried out according to the manufacturer's instruction. The efficiency of siRNA interference was examined with Real-time PCR 48 hours later and with Western blot 72 hours later.

The article "Immunoglobulin G Expression in Lung Cancer and Its Effects on Metastasis" was retracted in 2020. Reasons: duplicated images; concerns about the results or conclusions.

### MTS assay

About 1×10^4^ cancer cells (A549 or SK-MES-1) were seeded and cultured on a 96-well plate for 24 h. The cells were divided into the following groups: treated groups (siRNA-scrambled and siRNA-IGHG1), untreated group and blank group (complete medium without cancer cell). The RNA interference procedure was carried out and cultured for a 48-hour period. MTS (Jianchen Biosciences, Nanjing, China, 20 µl) was added to each well, and after incubation in a 5% CO_2_ atmosphere at 37°C for 1 h, the OD value of each well was read at 450 nm wavelength ultraviolet. The experiments were performed in triplicate. The cell proliferation was calculated as follows:


### Attachment assay

Details of attachment assays were described previously with minor modifications [37]. Briefly, the cultured A549, SK-MES-1 and Beas2B cells were transfected with siRNA. Two days later, 1×10^4^ cells per well were seeded on matrigel-coated 96-well plates (BD Biosciences, Franklin Lakes, NJ). After 2 hours, the plates were washed to remove non-adhesive cells. Each well was incubated with 20 µl MTS reagents for 2 hours at 37°C and the optical density was detected at 450 nm wavelength ultraviolet. Controls with scrambled siRNAs were performed with the same protocol described above. The cell seeding density is an empirical value. The aim is to establish 30% ∼50% cell confluence after cell adherence to the culture plate to facilitate growth. Once established, the seeding density was identical for all groups to ensure fair comparison.

### Transwell assay

Melted metrigel was mixed with precolled DMEM at a final concentration of 0.8 µg/µl and then coated on the upper chambers of transwell inserts (Millipore, Billerica, MA) at 100 µl/well until coagulating at 37°C. After 48 h of siRNA transfection, about 1×10^5^ trypsinized cells were seeded into the upper chamber using serum-free DMEM. Again, the cell seeding density was identical for all groups. The transwell inserts were set into 24-well plate wells in which 200 µl DMEM plus 10% FBS was placed. The plate was set still at 37°C for 24 h. Assays were then stopped by removing non-invading cells in the upper chamber with swabs. Cells in the lower side of the insert were stained with Hematoxylin. Cells in five visual fields under 400×magnification per insert were counted and photographed.

The article "Immunoglobulin G Expression in Lung Cancer and Its Effects on Metastasis" was retracted in 2020. Reasons: duplicated images; concerns about the results or conclusions.

### Wound healing assay

The cultured A549, SK-MES-1 and Beas2B cells seeded in 12-well plates (1×10^5^ cells/well) were transfected with siRNA as described above. When cells reached 90% confluency, erasing the cell monolayer with a sterile 10 µl pipette tip was used to create a wound area. Then, the plates were washed with PBS to remove detached cells, and cells were cultured with FBS-free DMEM. Subsequently, the plate was set still at 37°C for 48 h. The wound area was monitored with an inverted microscope and photographed.

### Statistical analysis

Correlations between Igγ expression in lung cancers and different clinical pathological parameters were performed with the Pearson chi-square test.

Student's t test was used to compare data obtained with the three groups, i.e. siRNA-IGHG1, siRNA-scrambled and the untreated in assays of MTS, transwell, attachment, Real-time PCR and Western blot. The correlations between Igγand MTA1 expressions and between MTA1 expression and clinical pathological parameters were evaluated with Student's t test. The level of significance was set at *p*<0.05.

## Results

### Igγ, Igκ and Igλ expressions in LSCC and LAC

Most lung cancers (>85%) examined expressed Igγ and Igκ, while a small number (<15%) also expressed Igλ at the same time. Igγ, Igκ and Igλ were expressed in the same cells as demonstrated with consecutive sections. Positive staining signals were localized to the cytoplasm and on the cellular membranes. The majority of positive cancer cells were distributed at the peripheral regions of the cancer nests in LSCC or with a discontinuous spotted pattern in the tubular structures of LAC (Figure 1, **A–F**). Many IgG postive cancer cells had atypical nuclei and nuclear condensation. Autopsied tonsils contained Igγ, Igκ and Igλ immunoreactivities in B lymphocytes (Figure 1, **G–I**). We utilized CD20 as a marker for B lymphocytes and pan CK as a marker for cells of epithelial origin. With serial sections, we detected two kinds of cells expressing Igγ. One is large epithelioid cells with positive pan CK, and the other is small round cells with positive CD20. Based on morphology and cell markers, we identified that the former are cancer cells and the latter are infiltrating B lymphocytes (Figure 1, **J–O**). Normal lung tissue adjacent to the cancer nests contained no positive IgG immunoreactivity (Figure 1, **P–R**).

**Figure 1:** IgG expression in LSCC and LAC with IHC. **A–C**, Igγ (**A**), Igκ (**B**) and Igλ (**C**) immunostainings are positive in the cytoplasm and cellular membrane of LSCC on serial sections. Note: The IgG positive cancer cells are distributed at the periphery of the tumor mass. **D–F**, positive signals for Igγ (**D**), Igκ (**E**) and Igλ (**F**) are shown in the cytoplasm and cellular membrane of a LAC. **G–I**, Igγ (**G**), Igκ (**H**) and Igλ (**I**) expressions are detected in lymphocytes of tonsil tissues as a positive control. **J–L**, Igγ (**J**), pan CK (**K**) and CD20 (**L**) are expressed in LSCC on serial sections. **M–O,** Igγ (**M**), pan CK (**N**) and CD20 (**O**) are expressed in serial sections of LAC. Igγ(**P**), Igκ (**Q**) and Igλ (**R**) are not expressed in normal epithelial cells adjacent to tumor mass on serial sections. Black arrowheads point to the same cancer cell on serial sections. Black arrows point to positive lymphocytes. With AEC colorization, the positive immunostainings with AEC are red in color. Note: IgG is positive in both cancer cells and infiltrating lymphocytes with the latter stronger than the former. Scale bar: 20 µm.

The article "Immunoglobulin G Expression in Lung Cancer and Its Effects on Metastasis" was retracted in 2020. Reasons: duplicated images; concerns about the results or conclusions.

In the antibody pre-absorption tests, increasing concentrations of pure human IgG antigen led to decreasing intensity of immunostaining (Figure 2, **A–F**). Infiltrating B lymphoctyes in the mesenchyma surrounding the cancer nests or the tubular structures expressed IgG stronger than that of the cancer cells. To further distinguish cancer cells from lymphocytes, we examined the expressions of CD16, CD32, CD64 and FcRn in LSCC and LAC. No cancer cells were found to express these receptors (Figure 3, **A–H**) and the only cells expressing them were lymphocytes (Figure 3, **I–L**).

**Figure 2:** Igγ Antibody preabsorption tests in LSCC and LAC. **A–C**, the mouse anti-human Igγ monoclonal antibody: pure human IgG  = 1∶1, 1∶5, and 1∶10 in LSCC sections. **D–F**, the similar gradient ratio of Igγ: pure human IgG in LAC sections. With the increase of antigen concentration (pure human IgG), the positive IgG signal was weakened. Bar: 20 µm.

**Figure 3:** Receptors for Igγ were not expressed on the cellular membrane of lung cancer cells. CD16 (Fcγ receptor III) is shown in LSCC (**A**) and LAC (**E**) tissues. CD32 (Fcγ receptor II) is displayed in LSCC (**B**) and LAC (**F**) tissues. CD64 (Fcγ receptor I) is shown in LSCC (**C**) and LAC (**G**) tissues. FcRn (neonatal Fcγ receptor) is shown in LSCC (**D**) and LAC (**H**) tissues. In those sections, positive signals are only expressed in the cytoplasm and membrane of lymphocytes, while no positive signals are found in cancer cells. CD16 (**I**), CD32 (**J**), CD64 (**K**) and FcRn (**L**) are expressed in biopsied human tonsil tissues as positive controls. Bar: 20 µm.

Almost all cancer cells were positive for IGHG1 mRNA. In consecutive sections, the protein of Igγ and mRNA of IGHG1 were localized to the cytoplasm of the same cancer cells and infiltrating B lymphocytes (Figure 4, **A, B, D** and **E**). Positive signals of IgG mRNA were also found in B lymphocytes of human tonsil tissues (Figure 4, **G** and **H**). No positive signal was seen in lymphocytes and cancers when the sense probe was used (Figure 4, **C, F** and **I**). Normal lung tissue adjacent to the cancer nests did not express IgG protein and mRNA of IGHG1 (Figure 4, **J–L**).

The article "Immunoglobulin G Expression in Lung Cancer and Its Effects on Metastasis" was retracted in 2020. Reasons: duplicated images; concerns about the results or conclusions.

**Figure 4:** IgG expression in lung cancer tissue with IHC and ISH. Colocalization of the IgG mRNA and protein in LSCC and LAC tissue samples demonstrated with ISH and IHC. **A–C**, Igγ immunostaining (**A**, red) and mRNA signals (**B**, purple, with antisense probe) are positive on serial sections of a LSCC. **C** is a negative control with sense probe. **D–F**, Igγ immunostaining (**D**, red) and mRNA signals (**E**, purple, with antisense probe) are positive on serial sections of a LAC. **F** is negative with sense probe. **G–I**, Tonsil tissues are used as a positive control. **G** is for Igγ with IHC showing positive lymphocytes. **H** is for the antisense probe with ISH showing positive lymphocytes. **I** is with sense probe in ISH showing no positive signal. **J–L**, Igγ protein (**J**) and mRNA (**K**, the antisense probe) are not expressed in normal epithelial cells adjacent to tumor mass. **L** is the sense probe. Black arrowheads point to the same cancer cells on serial sections. Black arrows point to positive lymphocytes.

With fresh surgical lung cancer tissue, we performed LMD to capture cancer cells and normal lung epithelial cells adjacent to cancer nests only without lymphocytes (Figure 5, **A**) to detect the mRNA transcripts of IgG including IGHG1, κ constant (Cκ), λ constant (Cλ), γ variable (Vγ), κ variable (Vκ), λ variable (Vλ), sterile germ line transcripts (Iγ-Cγ) and essential enzymes including RAG1, RAG2 and AID for immunoglobulin synthesis and class switching. Positive signals of these genes were found in LSCC and LAC cancer cells instead of normal lung epithelial cells (Figure 5, **B**). Four cases of lung cancers showed very high homology to the published sequences of Vγ, Vκ, and Vλ only with few gene mutations. By sequence alignment, we also found that the V (D) J rearrangement occurred when the heavy chain or light chains were synthesized, but presented a monotonous pattern (Figure 6).

**Figure 5:** IgG expression in lung cancer tissue with LMD coupled with RT-PCR. **A** is the representative photos of LMD in LSCC, LAC and normal lung adjacent to tumor mass. **B**, the bands represented that IgG synthesis associated genes were detected in LSCC, LAC and normal lung with LMD coupled with RT-PCR. No CD19 was detected, thereby excluding possible B lymphocyte contamination. Raji cell line was used as a positive control. Water was used as a negative control in place of the primers. RNA treated with DNase (abbreviated as R) was used as a template to exclude possible false positivity in 1R-6R. NL is the abbreviation of normal lung.

The article "Immunoglobulin G Expression in Lung Cancer and Its Effects on Metastasis" was retracted in 2020. Reasons: duplicated images; concerns about the results or conclusions.

**Figure 6:** The sequencing results of IgG mRNA extracted from LSCC and LAC. **A** is for the sequences of Vγ, **B** is for Vκ, and **C** is for Vλ.

### Detection of IgG and the essential enzymes for IgG synthesis in A549, SK-MES-1 and Beas2B cell lines

LSCC cell line (SK-MES-1) and LAC cell line (A549) were found to express Igγ, Igκ and Igλ with immunofluorescence (Figure 7, **A–F**). The positive signal was seen in the cytoplasm and on cell membrane. As a positive control, Igγ, Igκ and Igλ were also detected in the cytoplasm of Raji cells (Figure 7, **G–I**). Normal lung epithelial cell line (Beas2B) did not express Igγ, Igκ and Igλ (Figure 7, **J–L**). Abundant IGHG1 mRNA was detected in A549 and SK-MES-1 (Figure 7, **M** and **O**) as well as Raji cells (Figure 7, **Q**). No positive signal was seen when sense probe was used (Figure 7, **N**, **P** and **R**). IGHG1 mRNA was not found in Beas2B (Figure 7, **S** and **T**).

**Figure 7:** IgG expression in lung cancer cell lines with ISH and immunofluorescence. **A–C**, Igγ (**A**), Igκ (**B**) and Igλ (**C**) are expressed in A549 cells with immunofluorescence. **D–F**, Igγ (**D**), Igκ (**E**) and Igλ (**F**) are expressed in SK-MES-1 cells. **G–I**, Igγ (**G**), Igκ (**H**) and Igλ (**I**) are in Raji cells as positive control. **J–L**, Igγ (**J**), Igκ (**K**) and Igλ (**L**) are not expressed in Beas2B cells. Positive signals (purple) for IGHG1 antisense probe are seen in the cytoplasm of A549 (**M**), SK-MES-1 (**O**) and Raji (**Q**) cells. **N**, **P** and **R** show negative results (sense probe) in A549, SK-MES-1 and Raji cells. No positive signals are found in Beas2B cells (**S**, the antisense probe; and **T**, the sense probe). To highlight the cells without purple signal, methyl green was use to counterstain the nuclei. Scale bars: 20 µm.

The mRNAs of IgG and the essential enzymes for IgG synthesis were all expressed in A549 and SK-MES-1 instead of Beas2B (Figure 8, **A**). The whole molecule of IgG as well as different fragments, i.e. Igγ, Igκ and Igλ were all detectable in A549 and SK-MES-1 cells (Figure 8, **B**) with corresponding molecular weight similar to IgG from B lymphocytes. The presence of RAG1, RAG2 and AID in A549 and SK-MES-1 was also confirmed with Western blot (Figure 8, **C**). Contrary to the cancer cells, Beas2B did not express IgG components or those enzymes for IgG synthesis (Figure 8, **B** and **C**).

The article "Immunoglobulin G Expression in Lung Cancer and Its Effects on Metastasis" was retracted in 2020. Reasons: duplicated images; concerns about the results or conclusions.

**Figure 8:** IgG expression in lung cancer cell lines with RT-PCR and Western blot. **A**, the bands represented that IgG synthesis associated genes were detected with RT-PCR in A549 and SK-MES-1, whereas not in Beas2B. **B** shows that IgG whole molecule, Igγ, Igκ and Igλ are detected in A549, SK-MES-1, whereas not in Beas2B with Western blot. Human pure IgG was used as molecular weight standard to compare with that from lung cancer cells. Raji cell line was a positive control. **C** shows that RAG1, RAG2 and AID are expressed in lung cancer cells, whereas not in Beas2B. Raji cell line was served as a positive control.

### IgG and MTA1 gene expressions were inhibited by siRNA interference to IGHG1

The expression of Igγ at both mRNA (Figure 9, **A**) and protein levels (Figure 9, **C** and **D**) were specifically down-regulated by siRNA-IGHG1 in A549 and SK-MES-1cell lines. Along with IgG, MTA1 expression was markedly decreased at the mRNA (Figure 9, **B**) and the protein levels (Figure 9, **C** and **D**) in the two cell lines. The differences between siRNA-IGHG1 and the two other control groups were statistically significant (*p*<0.05).

**Figure 9:** IgG expression was strongly correlated to MTA1 expression and IgG down-regulation lowered MTA1 expression. **A**, IgG was down-regulated with specific IGHG1 siRNA transfection with Real-time PCR. **B**, MTA1 expression was lowered following the decrease of IgG expression detected with Real-time PCR. **C**, typical bands represent the changes of IgG and MTA1 expressions after IGHG1 siRNA interference in A549 cell line. **D**, similar changes in SK-MES-1 cell line. **E**, Igγ (red, positive staining in cytoplasm) was mostly co-localized with MTA1 (purplish red, positive staining in nuclei) in lung cancers. Black arrows or arrowheads show typical cancer cells labeling with IgG and MTA1. **F**, lung cancers with weak IgG expression have a lower expression level of MTA1 in comparison to strong IgG expression cancers. **G**, lung cancers with lymph node metastasis have much higher MTA1 expression than non-metastatic cancers. The histograms represent the four independent assays. Data are presented as mean ± S.E. *, *p*<0.05. Scale bars: 20 µm.

### Down-regulation of IgG expression with siRNA interference inhibited the proliferation of lung cancer cells

As shown in Figure S1, lung cancer cell proliferation was decreased by over 50% in the siRNA-IGHG1 treated group. The differences between siRNA-IGHG1 and the two other control groups were statistically significant (*p*<0.05). The proliferation ratio in the group of siRNA-scrambled was not significantly different from that of the untreated group (*p*>0.05) suggesting that transfection reagent had low toxicity to cell proliferation.

The article "Immunoglobulin G Expression in Lung Cancer and Its Effects on Metastasis" was retracted in 2020. Reasons: duplicated images; concerns about the results or conclusions.

### Correlation between Igγ expression and clinical and pathological parameters

Among 86 lung cancer specimens, 66 (76.74%) expressed Igγ with 20/86 (23.26%), 21/86 (24.42%), 21/86 (24.44%) and 24/86 (27.96%) cases showing −, +, ++, and +++ scores, respectively (Table 1). Statistical analysis unveiled that Igγ expression was associated to histological grade, clinical stage and lymph node metastasis, but not to sex and age of the patients (Table 1). For IgG-positive cancer cells, the positive rate of MTA1 was 75.43%, while for MTA1-positive cancer cells, the positive rate of IgG was 77.29%. MTA1 was mostly co-localized with IgG (Figure 9, **E** and **F**). It is also correlated to histological grade, clinical stage and lymph node metastasis ((Figure 9, **G**) with statistical significance.

**Table 1:** Statistical analysis for Igγ immunoreactivity intensity and clinicopathological parameters in 86 lung squamous cell carcinomas and adenocarcinomas.

Variable	No. of samples for Igγ immunoreactivity intensity scores				Total	?^2^	*p*
	−	+	++	+++			
Sex							
Male	9	13	11	14	47	1.37	0.712
Female	11	8	10	10	39		
Ages (y)							
≤55	10	6	7	9	32	2.21	0.529
>55	10	15	14	15	54		
Histological type							
LSCC	9	12	13	12	46	1.41	0.703
LAC	11	9	8	12	40		
Tumor stage							
I	10	12	4	3	29	23.82	<0.01
II	7	4	14	8	33		
III-IV	3	5	3	13	24		
Pathological grade							
WD	13	12	5	5	35	22.2	<0.01
MD	4	7	11	6	28		
PD	3	2	5	13	23		
Lymph node metastasis							
Yes	7	7	15	17	46	11.6	<0.05
No	13	14	6	7	40		

Scored as −, negative; +, weak; ++, moderate; and +++, strong.

Abbreviation: LSCC, lung squamous cell carcinoma; LAC, lung adenocarcinoma; WD, well differentiated; MD, moderate differentiated; PD, poor differentiated.

### Down-regulation of IgG expression with siRNA interference inhibited cancer cell migration and attachment

In comparison to the untreated group and the siRNA-scrambled group, siRNA treatment against IGHG1 mRNA sequence reduced the ability of migration and attachment of lung cancer cells (Figure 10, **A** and **B**). The differences between siRNA IGHG1 treated and the two other control groups were statistically significant in the migration and the attachment assays (*p*<0.05). Results of the wound healing assay were similar to that of the transwell assay, showing that with inhibition of IgG expression in cancer cells, the ability of healing repair was reduced (Figure 11). On the contrary, with siRNA treatment, normal lung epithelial cells did not decrease the ability of healing repairment (Figure 10, **A** and **B**).

The article "Immunoglobulin G Expression in Lung Cancer and Its Effects on Metastasis" was retracted in 2020. Reasons: duplicated images; concerns about the results or conclusions.

**Figure 10:** IgG down-regulation inhibits lung cancer cell migration and attachment. With specific IGHG1 siRNA transfection, the ability of migration and attachment of lung cancer cells was reduced markedly in A549 and SK-MES-1 cells, whereas not in Beas2B cells. **A**, representative photographs (200×) of transwell assays. **B**, representative photographs (200×) of attachment assays. The histograms represent the four independent assays. Data are presented as mean ± S.E. *, *p*<0.05.

**Figure 11:** IgG down-regulation inhibits cell migration by wound healing assay in lung cancer cells. Forty-eight hours after scratching the cultured cells, scratched areas were photographed. The results show that for the untreated and siRNA-scrambled groups, the wound area is markedly narrowed in A549 and SK-MES-1 but not in Beas2B.

### With siRNA interference to MTA1, the ability of migration and attachment reduced in cancer cells, whereas did not change in normal lung cells

With siRNA interference to MTA1 mRNA, we found that MTA1 expression was markedly reduced compared with the untreated group and the siRNA-scrambled group in A549 and SK-MES-1(Figure S2, **A** and **B**). Along with the change of MTA1 expression, the ability of migration and attachment was markedly inhibited in A549 and SK-MES-1(Figure S3, **A** and **B**; Figure S4). The differences of MTA1 expression, migration and attachment between siRNA-MTA1 treated and the two other control groups were statistically significant (*p*<0.05). Contrary to A549 and SK-MES-1, MTA1 was weakly expressed in Beas2B and was not influenced by siRNA interference (Figure S2, **C**). The ability of migration and attachment was not affected by siRNA treatment in the assays of transwell, attachment and wound healing (Figure S3, **A** and **B**; Figure S4).

## Discussion

In this study, we established the ability of lung cancer cells and related cell lines to express IgG gene. To ensure that IgG was synthesized by lung cancer cells, but not absorbed from the surroundings, we detected abundant IgG mRNA as well as gene expression of the essential enzymes for IgG synthesis, RAG1, RAG2 and AID in lung cancer cells. LMD coupled with RT-PCR further confirmed the ability of lung cancer cells to synthesize IgG. The possible contamination of other cell types, particularly lymphocytes and plasma cells, in the tested samples was ruled out with corresponding cell markers and laser dissection which isolated cancer cells only. In addition, we did not find IgG receptor molecules CD16, CD32, CD64 or FcRn in lung cancer cells, further excluding possible phagocytosis and internalization of IgG by cancer cells [38], [39]. Furthermore two lung cancer cell lines were found to contain IgG protein immunoreactivity and IgG mRNA. Transfer of IgG mRNA and protein from B lymphocytes to cancer cells by exosomes can be ruled out. Therefore the IgG we detected in lung cancer cells were synthesized by these cells but not absorbed from the serum or surrounding tissue. In normal lung epithelial cells and a related cell line, we did not find expressions of IgG genes and related essential enzymes for its synthesis with immunohistochemistry, ISH, immunofluorescence and RT-PCR. These observations showed that IgG derived from lung cancer cells was likely a product of epithelial malignant transformation.

The article "Immunoglobulin G Expression in Lung Cancer and Its Effects on Metastasis" was retracted in 2020. Reasons: duplicated images; concerns about the results or conclusions.

Previously, at least 8 groups from five countries have independently found IgG production by cancer cells, but IgG expression in lung cancer has been mentioned only sporadically on a small number of cases [5], [6], [40]. A systematic study on large cohorts of lung cancer patients has not been available and the effects of lung cancer-produced IgG on cancer cell behavior have not been investigated. In this study, we found that the extents of IgG expression in 86 lung cancers were positively related to clinical stage, pathological grade and lymph node metastasis. We also found that IgG of cancerous origin has the ability of promoting growth and survival of tumor cells. The fact that Western blot and IHC with antibodies raised against classic IgG, which was extracted from B lymphocytes and plasma cells, detected IgG in lung cancer cells suggests that cancerous IgG has similar antigenic epitopes to that synthesized by B lymphocytes and plasma cells. We also demonstrated that different parts of IgG gene was transcripted in lung cancer cells, suggesting that cancerous IgG may have similar mRNA structures to that of B lymphocytes and plasma cells. However, the functions of the two IgGs appeared quite different. A possible explanation is that IgG of cancerous origin has chemical modification that is different from that of B lymphocytes. Taylor et al found an immunoglobulin molecule in ovarian cancers with strong glycosylation that had a significant correlation with malignant grades of the cancers [41], [42]. Lee et al. found CA215, an immunoglobulin superfamily protein, with a unique carbohydrate-associated epitope and a similar ability to promote cancer cell progression [24], [43]. Therefore, it is possible that the IgG we detected from the cancer cells were the same or similar to those previously reported IgG-like proteins in cancer cells but different from that produced by B lymphocytes or plasma cells.

In this study, we found that almost all the cancer cells were positive for IGHG1 mRNA, whereas only some of these cells were positive for IgG immunostaining. This phenomenon could be caused by posttranscriptional modification. It is common that mRNA distribution is more extensive than protein expression for a given gene. We also observed that IgG was mainly distributed in the periphery of the cancer nests in LSCC and had discontinuous spotted expression pattern in the tubular structures of LAC. Moreover, the IgG postive cancer cells had atypical nuclei and nuclear condensation. We also found that lung cancers with lymph node metastasis had higher expression rate of IgG. Similar observations were made by Ma et al in breast cancers [29]. These observations suggest that IgG producing cancer cells may have disordered cell cycles and chromatin replication. Based on the above and the results of our functional assays, it is likely that the IgG positive cells distributed at the periphery of the cancer nests in LSCC and discontinuously in the tubular structures of LAC are the cell population prone to metastasize and survive at distant sites. These cells would triumph over IgG negative cancer cells and eventually metastasize. The positive relationship between IgG and clinical parameters gives raise to the possible role for IgG as a prognostic marker.

The article "Immunoglobulin G Expression in Lung Cancer and Its Effects on Metastasis" was retracted in 2020. Reasons: duplicated images; concerns about the results or conclusions.

We also attempted to elucidate the molecular mechanism of IgG expression in metastasis. With the technique of siRNA interference, we inhibited the IgG expression in two lung cancer cell lines. Subsequently, migration, attachment and wound healing assays, which simulated important behavior of cancer cell during metastasis, were also inhibited along with the decrease of IgG synthesis, suggesting that cancerous IgG may influence the ability of metastasis of lung cancer. Moreover, in normal lung epithelial cells which did not express IgG, siRNA interference to IGHG1 gene expressoin did not change their ability of migration and attachment, further confirming the role of IgG in cancer cell metastasis. Recently, Pelegrina et al reported that IgG from blood of breast cancer patients in T1N0Mx stage promoted cancer cell proliferation and migration [44], [45]. These reports support our findings in lung cancer and our previous report on the functions of cancerous IgG [46]. Following siRNA treatment to down-regulate IgG gene expression in the two lung cancer cell lines, we tested a range of common metastatic related genes including CD44, E-cadherin, MMP9, MMP2, Intergrin-β1 and MTA1with Real-time PCR and Western blot. Only MTA1 showed significant suppression after inhibiting IgG expression in A549 and SK-MES-1 cell lines. The significant co-localization of MTA1 and IgG suggests that there might be a relationship between IgG and MTA1 in regulating the behavior of lung cancers. MTA1 is known to regulate the transcription of metastasis-related genes by modifying the target chromatin acetylation status as well as cofactor accessibility to the target DNA. High MTA1 expression was strongly associated with invasion and lymphatic metastasis in various carcinomas [32], [33], [47]. With siRNA interference to MTA1, MTA1 expression in lung cancer cells was markedly decreased which in turn inhibited the ability of migration and attachment. As a control, normal lung epithelial cells were not influenced in the same assays. This finding indicates that cancer-derived IgG might exert its effect via MTA1 signaling pathway in lung cancer and has the potential to be a target for cancer therapy.

The article "Immunoglobulin G Expression in Lung Cancer and Its Effects on Metastasis" was retracted in 2020. Reasons: duplicated images; concerns about the results or conclusions.

In conclusion, we demonstrated that IgG can be produced by lung cancer cells. IgG expression in lung cancer cells is closely related to clinical stage, pathological grade and lymph node metastasis, making IgG a potential clinical prognostic indicator for lung cancer. In addition, the findings obtained with functional assays and IgG siRNA down-regulation suggest that cancerous IgG may play a key role in lung cancer growth and metastasis through regulating the metastatic gene MTA1, thus providing new clues for the treatment of lung cancer.

## Supporting Information

Figure S1 **IGHG1 siRNA induced reduction of IgG expression inhibited lung cancer cell proliferation.** A, A549 cell line. B, SK-MES-1 cell line. The histograms represent the three independent assays. Data are presented as mean ± S.E. *, p<0.05.
(DOCX)

Figure S2 **MTA1 was down-regulated with specific MTA1 siRNA transfection with Western blot.** A, typical bands represent the changes of MTA1 expression after MTA1 siRNA interference in A549 cell line. B, the similar changes in SK-MES-1 cell line. C, MTA1 is weakly expressed in Beas2B and is almost not influenced after siRNA interference to MTA1. The histograms represent the four independent assays. Data are presented as mean ± S.E. *, p<0.05. Scale bars: 20 µm.
(DOCX)

Figure S3 **MTA1 down-regulation inhibits lung cancer cell migration and attachment.** With specific MTA1 siRNA transfection, the ability of migration and attachment of lung cancer cells was reduced markedly in A549 and SK-MES-1 cells, whereas not in Beas2B cells. A, representative photographs (200×) of transwell assays. B, representative photographs (200×) of attachment assays. The histograms represent the four independent assays. Data are presented as mean ± S.E. *, p<0.05.
(DOCX)

Figure S4 **MTA1 down-regulation inhibits cell migration by wound healing assay in lung cancer cells.** Forty-eight hours after scratching the cells, scratched areas were photographed. The results show that for the untreated and siRNA-scrambled groups, the wound area is markedly narrow in A549 and SK-MES-1 than that in Beas2B.
(DOCX)

Table S1 **Antibodies used in this study.**
(DOCX)

Table S2 **Primers used in RT-PCR and LMD coupled with RT-PCR.**
(DOCX)

Table S3 **Primers used in Realtime PCR.**
(DOCX)
